# Long non-coding RNA-ROR aggravates myocardial ischemia/reperfusion injury

**DOI:** 10.1590/1414-431X20186555

**Published:** 2018-04-23

**Authors:** Weiwei Zhang, Ying Li, Peng Wang

**Affiliations:** 1 Department of Cardiology, Dezhou People's Hospital, Dezhou, China; 2 Interventional Center, Dezhou People's Hospital, Dezhou, China

**Keywords:** lncRNA, Ischemia/reperfusion (I/R), Hypoxia/reoxygenation (H/R), Cell viability, Apoptosis

## Abstract

Long non-coding RNAs (lncRNAs) play an important role in the pathogenesis of cardiovascular diseases, especially in myocardial infarction and ischemia/reperfusion (I/R). However, the underlying molecular mechanism remains unclear. In this study, we determined the role and the possible underlying molecular mechanism of lncRNA-ROR in myocardial I/R injury. H9c2 cells and human cardiomyocytes (HCM) were subjected to either hypoxia/reoxygenation (H/R), I/R or normal conditions (normoxia). The expression levels of lncRNA-ROR were detected in serum of myocardial I/R injury patients, H9c2 cells, and HCM by qRT-PCR. Then, levels of lactate dehydrogenase (LDH), malondialdehyde (MDA), superoxide dismutase (SOD), and glutathione peroxidase (GSH-PX) were measured by kits. Cell viability, apoptosis, apoptosis-associated factors, and p38/MAPK pathway were examined by MTT, flow cytometry, and western blot assays. Furthermore, reactive oxygen species (ROS) production was determined by H2DCF-DA and MitoSOX Red probes with flow cytometry. NADPH oxidase activity and NOX2 protein levels were measured by lucigenin chemiluminescence and western blot. Results showed that lncRNA-ROR expression was increased in I/R patients and in H/R treatment of H9c2 cells and HCM. Moreover, lncRNA-ROR significantly promoted H/R-induced myocardial injury via stimulating release of LDH, MDA, SOD, and GSH-PX. Furthermore, lncRNA-ROR decreased cell viability, increased apoptosis, and regulated expression of apoptosis-associated factors. Additionally, lncRNA-ROR increased phosphorylation of p38 and ERK1/2 expression and inhibition of p38/MAPK, and rescued lncRNA-ROR-induced cell injury in H9c2 cells and HCM. ROS production, NADPH oxidase activity, and NOX2 protein levels were promoted by lncRNA-ROR. These data suggested that lncRNA-ROR acted as a therapeutic agent for the treatment of myocardial I/R injury.

## Introduction

Myocardial ischemia/reperfusion (I/R) injury leads to adverse cardiovascular outcomes following myocardial ischemia, cardiac surgery or circulatory arrest and is one of the major causes of morbidity and mortality in humans with coronary heart disease (1). The pathology of the disease suggests that myocardial infarction and angina pectoris are accompanied by changes in gene expression (2). The underlying molecular mechanisms of myocardial I/R injury are complex and include oxidative stress, intracellular Ca^2+^ overload, rapid restoration of physiological pH upon reperfusion, mitochondrial permeability transition pore, and exaggerated inflammation (3). Rapid alterations in ion flux and renormalization of pH following reperfusion causes severe cytotoxicity and I/R injury, characterized by cell death and functional deterioration because of restoration of blood flow (4). I/R injury causes local myocardial inflammation and apoptosis, which in turn leads to irreversible damage to the myocardium. However, early restoration of blood flow through the occluded coronary artery might reduce mortality by limiting the infarct size and preserving cardiac function (5,6). Despite restoration of blood flow, reperfusion alone seems not to be enough to save the myocardium because of the complications that arise from the loss of viability (7).

Following myocardial I/R injury, there is a sudden increase in cytokines and chemokines and influx of leukocytes into the endangered myocardial region (8). Cell survival and extracellular matrix integrity by activation of pro-apoptotic signaling pathways (including mitogen-activated protein kinases and p38) are hampered by inflammatory responses after myocardial I/R injury (9). Studies indicate that cell death is a key factor in the pathogenesis of various cardiac diseases such as heart failure, myocardial infarction, and I/R injury (1). During heart disease, myocytes are lost due to both apoptosis and necrosis (10). It suggests that necrosis plays a critical role in the pathogenesis of the cardiac disease (11). However, the underlying mechanism of cardiomyocyte death is still not clear. Thus, I/R injury is still a major problem in the treatment of myocardial ischemia.

Long non-coding RNAs (lncRNAs) belong to a newly discovered class of genes in the human genome that have been proposed to be key regulators of biological processes (12). lncRNAs consist of more than 200 nucleotides (13). Recent evidence shows that lncRNAs play an important role in the physiological processes such as differentiation, proliferation, apoptosis, and inflammation (14). It is also observed that lncRNAs are highly regulated and specific (15). However, the role of lncRNA-ROR in myocardial I/R injury remains unclear.

The objective of this study was to investigate the role and the possible underlying molecular mechanism of lncRNA-ROR in myocardial I/R injury. This study will provide a new insight for the treatment of cardiomyocytes injury.

## Material and Methods

### Serum samples

Serum samples of 20 normal individuals and 20 patients with myocardial I/R injury were obtained from Dezhou People's Hospital. The study was approved by the Research Ethics Committee of Dezhou People's Hospital, and written informed consent was obtained from all participants. The samples were collected and frozen in liquid nitrogen, and stored at −80°C.

### Cell culture and H/R exposure

Embryonic rat myocardium-derived cells H9c2 and human cardiomyocytes (HCM) were purchased from the American Type Culture Collection (ATCC, USA) and cultured in Dulbecco's Modified Eagle's Medium (DMEM; Sigma, USA) containing 10% fetal calf serum (FCS; Invitrogen, USA) (16). In brief, H9c2 cells and HCM in serum-free DMEM were placed in a humidified chamber equilibrated with 5% CO_2_ and 95% N_2_ for 4 h, followed by reoxygenation with 5% CO_2_ and 95% air for 3 h in DMEM with 10% FCS. Hypoxia/reoxygenation (H/R) treatment of H9c2 cells and HCM were performed as described previously. Gene expression and apoptotic changes were measured at 24 h after re-oxygenation. Cells cultured under normoxic conditions were used as control.

### Cell transfection

Small interfering RNAs (siRNAs) targeting mRNA (si-lncRNA-ROR) and pcDNA3.1-lncRNA-ROR (lncRNA-ROR) were synthesized by RiboBio (China). Transfections were performed in 6-, 24-, or 96-well plates after seeded cells were cultured for 24 h. All transfections were done with HiPerFect transfection reagent (QIAGEN, Germany) according to the manufacturer's protocol. Briefly, 5×10^3^ cells/cm^2^ were seeded on 200 μL/cm^2^ culture. The siRNAs or pcDNAs were pre-incubated with HiPerFect transfection reagent at room temperature for 10 min. The complex was then transfected into the cardiomyocytes cells at a final concentration of 50 nM. The transfected cells were incubated under normal growth conditions for 48 h.

### Detection of LDH, MDA, SOD, and GSH-PX

Lactate dehydrogenase (LDH), malondialdehyde (MDA), superoxide dismutase (SOD), and glutathione peroxidase (GSH-PX) commercial kits were purchased from Sangon Biotech (China). The release levels of LDH, MDA, SOD, and GSH-PX were measured according to the manufacturer's instructions.

### Quantitative real-time PCR (qRT-PCR)

Total RNA was isolated using TRIzol reagent (Invitrogen), and complementary DNA (cDNA) was synthesized with PrimeScript reverse transcriptase (TaKaRa, China) and oligo-dT (20 bp) following the manufacturer's instructions. Reverse transcription PCR (RT-PCR) or real-time PCR was performed to analyze mRNA expression. The RT-PCR program was as follows: 94°C for 5 min, followed by 35 cycles of 94°C for 30 s, 50°C annealing for 30 s, and 72°C for 30 s. Real-time PCR was performed using SYBR Premix Ex TaqTM II kit (TaKaRa) as follows: 94°C for 10 s, followed by 40 cycles of 94°C for 5 s, 52°C for 30 s to anneal, and 72°C for 15 s. The relative level of lncRNA-ROR was determined using the 2^-ΔΔCt^ analysis method.

### Western blot analysis

Proteins were extracted from the primary cardiomyocytes in RIPA buffer (1% Triton X-100, 150 mmol/L NaCl, 5 mmol/L EDTA, and 10 mmol/L Tris-HCl, pH 7.0; Solarbio, China) supplemented with a protease inhibitor cocktail (Cat: I3786-1ML, Sigma). The cell lysates were separated by 10% sodium dodecyl sulfate-polyacrylamide gel electrophoresis (SDS-PAGE) and transferred electrophoretically to a PVDF membrane (Millipore Corporation, USA). After blocking with 8% milk in PBS, pH 7.5, the membranes were incubated with the following specific primary antibodies of Bax (ab32503), Bcl-2 (ab59348), cytochrome C (ab13575), Smac/Diablo (ab32023), cleaved-capase-3 (ab13847), cleaved-capase-9 (ab2324), p-p38 (ab47363), p38 (ab31828), p-ERK (ab214362), and ERK1/2 (ab196883; all at a dilution of 1:1000, Abcam, UK). After overnight incubation, the appropriate HRP-conjugated anti-rabbit IgG secondary antibody (ab205781, Abcam, all at a dilution of 1:5000) was subsequently applied and immunodetection was achieved using the ECL Plus detection system (Millipore Corporation) according to the manufacturer's instructions. Band intensity was quantified using Image Lab™ Software (Bio-Rad, China). GAPDH (ab8245, Abcam) was used as an internal control.

### Cell viability assay

To explore the effect of lncRNA on cell viability, 5000 cells per well in a 100 μL medium were seeded in 96-well plates. Every 24 h after transfection, 20 μL of the 3-(4,5-dimethylthiazol-2-yl)-2,5-diphenyltetrazolium bromide (MTT) reagent (Solarbio) was added to wells and incubated with these cells for 4 h. After removing the medium, blue formazan was dissolved with 200 μL dimethyl sulfoxide (DMSO; Sigma), and absorbance was measured at 570 nm. Wells containing only cardiomyocyte cells served as blanks.

### Cell apoptosis assay

To quantify apoptotic cells, flow cytometry was performed with an Annexin V-fluorescein-5-isothiocyanate apoptosis detection kit (Bio-vision, USA). After transfection for 48 h, cells were harvested in a 5-mL tube. Then, the cells were washed with cold PBS and re-suspended in 1×binding buffer (10 mM HEPES, 140 mM NaCl, 2.5 mM CaCl_2_, pH 7.4) at a final concentration of 1×10^6^ cells/mL. FITC-AnnexinV (5 μL) and propidium iodide (PI, 5 μL) were gently mixed and incubated with the cells for 15 min at room temperature. After incubation, the samples were analyzed by flow cytometry within 1 h.

### Measurement of reactive oxygen species (ROS) production

For examining the accumulation of intracellular ROS in H9c2 cells, the ROS assay kit purchased from Beyotime Institute of Biotechnology (Haimen, China) was used according to the manufacturer's instructions. Briefly, after treatment, cells were grown in a 96-well plate and incubated with 10 μmol/L of H2DCF-DA at 37°C for 1 h. The fluorescence intensity was measured using the fluorescence plate reader (BD Falcon, USA) at Ex./Em. = 488/525 nm.

### Measurement of mitochondrial ROS by MitoSOXRed

For detection of mitochondrial superoxide generation, MitoSOXRed assay (Invitrogen/Molecular Probes, USA) was performed. In brief, the treated H9c2 cells were incubated with 5 μM of MitoSOX Red for 30 min at 37°C. MitoSOX Red fluorescent intensity was determined at 510 nm excitation and 580 nm emission. After incubation, these cells were washed twice with PBS, trypsinized, resuspended, and immediately submitted to flow cytometry analysis.

### Measurement of NADPH oxidase activity

NADPH oxidase activity was detected by using the lucigenin-enhanced chemiluminescence method as previously described (17). Briefly, treated cells were washed in PBS and re-suspended in cold Krebs-HEPES buffer. Then, 300 μL cell suspensions were homogenized with 100 strokes in a Dounce homogenizer on ice, and aliquots of the homogenates were used immediately. Subsequently, 100 μL of homogenates were added to 900 μL of phosphate buffer, pH 7.0, containing 1 mM EGTA, 150 mM sucrose, 5 μM lucigenin, and 100 μM NADPH to start the reaction. Chemiluminescence was measured every 15 s for 10 min in a luminometer. A buffer blank (less than 5% of the cell signal) was subtracted from each reading. The differences between the values obtained before and after adding NADPH were calculated, and these data represented the activity of NADPH oxidase.

### Statistical analysis

Data are reported as means±SE. Differences between groups were compared by a one-way ANOVA using Graphpad prism software 6.0 (GraphPad Software, San USA). P<0.05 was considered to be statistically significant difference.

## Results

### lncRNA-ROR was highly expressed in myocardial I/R and H/R

Data indicated that the expression level of lncRNA-ROR was significantly increased by almost 2 times in the I/R group compared to the normal group (P<0.01, Figure 1A). In addition, lncRNA-ROR expression was increased by approximately 3 times in H9c2 cells and HCM after treatment of H/R compared to cells under normoxia (P<0.05, Figure 1B and C). These data suggested that lncRNA-ROR was highly expressed in myocardial I/R and H/R.

**Figure 1.** lncRNA-ROR was highly expressed in myocardial ischemia/reperfusion (I/R) and hypoxia/reoxygenation (H/R). *A*, Relative lncRNA-ROR expressions in serum of I/R injury patients and normal serum were detected by qRT-qPCR. *B*, and *C*, relative lncRNA-ROR expressions in H9c2 cells and human cardiomyocytes (HCM) after H/R treatment were also examined by qRT-PCR. Cells under normoxia served as the control group. Data are reported as means±SE. *P<0.05, **P<0.01 (ANOVA).

### lncRNA-ROR aggravated H/R-induced myocardial damage

H9c2 cells and HCM were assigned to normoxia, H/R, H/R+lncRNA-ROR, and H/R+si-lncRNA-ROR groups. The results showed that the level of LDH significantly increased after H/R treatment compared to control cells (P<0.01). Overexpression of lncRNA-ROR further increased LDH release by almost 31.5 and 38.2% in both H9c2 cells and HCM, respectively (P<0.01 or P<0.001), whereas, the promotive effect was obviously reversed by lncRNA-ROR inhibition (P<0.01) compared to H/R in H9c2 cells and HCM (Figure 2A).

**Figure 2.** Cells were assigned to normoxia, hypoxia/reoxygenation (H/R), H/R+lncRNA-ROR, and H/R+ASO-lncRNA-ROR groups. *A*, The release level of lactate dehydrogenase (LDH) and levels of (*B*) malondialdehyde (MDA), (*C*) superoxide dismutase (SOD), and (*D*) glutathione peroxidase (GSH-PX) in H9c2 cells and human cardiomyocytes (HCM) were evaluated by kits according to the manufacturer's instructions. H/R+lncRNA-ROR: H9c2 cells were transfected with lncRNA-ROR after H/R treatment. H/R+si-lncRNA-ROR: H9c2 cells were transfected with si-lncRNA-ROR after H/R treatment. Data are reported as means±SE. *P<0.05, **P<0.01, ***P<0.001 (ANOVA).

MDA is an important index of lipid peroxidation. As shown in Figure 2B, levels of MDA in H9c2 cells and HCM were significantly promoted after H/R treatment compared to control cells (P<0.001). As seen for LDH, lncRNA-ROR overexpression also increased MDA levels by 34.4 and 47.5% in H9c2 cells and HCM (P<0.05 or P<0.01), but suppression of lncRNA-ROR decreased MDA levels by 28.4 and 42.0% respectively, compared to the H/R group.

Levels of SOD and GSH-PX were significantly increased after treatment of H/R compared to the control group in H9c2 cells and HCM (Figure 2C and D). Moreover, lncRNA-ROR overexpression increased the levels of SOD and GSH-PX by 13.0 or 15.6% in H9c2 cells (P<0.05) and 28.6 or 13.2% in HCM, respectively (P<0.05), whereas, lncRNA-ROR suppression decreased by 21.9 or 19.7% in H9c2 cells (P<0.01) and 30.0 or 25.0% in HCM (P<0.05) compared to the H/R group.

### lncRNA-ROR aggravated H/R-induced cell injury by regulating cell viability and apoptosis

To explore the effect of lncRNA on cell viability, the cells were transfected with lncRNA-ROR and si-lncRNA-ROR for 24, 48, and 72 h. As shown in Figure 3A, cell viability at 24 h in normoxia, H/R, H/R+lncRNA-ROR, and H/R+si-lncRNA-ROR groups were 0.51, 0.36 (P<0.05), 0.26 (P<0.05), and 0.60 (P<0.05) in H9c2 cells and 0.47, 0.35 (P<0.05), 0.25 (P<0.05), and 0.46 (P<0.05) in HCM. MTT results showed that overexpression of lncRNA-ROR could further decrease the H/R-induced cell viability. We next observed the effect of lncRNA-ROR on cell apoptosis. The results showed that apoptotic cell rate in normoxia, H/R, H/R+lncRNA-ROR, and H/R+si-lncRNA-ROR groups were 17.8%, 23.4% (P<0.01), 28.7% (P<0.05), and 18.2% (P<0.05) in H9c2 cells and 4.4%, 14.6% (P<0.001), 18.1% (P<0.01), and 9.1% (P<0.01) in HCM. Flow cytometry showed that overexpression of lncRNA-ROR could further aggravate H/R-induced cell apoptosis (Figure 3B).

**Figure 3.** lncRNA-ROR aggravates hypoxia/reoxygenation (H/R)-induced cell injury by regulating cell viability and apoptosis. H9c2 cells and human cardiomyocytes (HCM) were transfected with lncRNA-ROR overexpression vector (lncRNA-ROR) and inhibition vector (si-lncRNA-ROR). After H/R treatment for 24 h, (*A*) cell viability, (*B*) apoptosis, and (*C*) and (*D*) apoptosis-related factors Bax, Bcl-2, cytochrome C, Smac/Diablo, cleaved-caspase-3, and cleaved-caspase-9 were measured by MTT, flow cytometry, qRT-PCR, and western blot, respectively. GAPDH served as the internal control. Data are reported as means±SE. *P<0.05, **P<0.01, ***P<0.001 (ANOVA).

To further explore the potential molecular mechanism of action of lncRNA-ROR, expression of apoptosis-related proteins such as Bax, Bcl-2, cytochrome C, Smac/Diablo, cleaved-caspase-3, and cleaved-caspase-9 were examined by qRT-PCR and western blot. Results revealed that H/R markedly increased Bax, cytochrome C, Smac/Diablo, cleaved-caspase-3, and cleaved-caspase-9 expressions, but decreased Bcl-2 expression. Overexpression of lncRNA-ROR further increased the expression of these five factors (P<0.05) and decreased the level of expression of Bcl-2 (P<0.01; Figure 3C and D). However, suppression of lncRNA-ROR showed a contrary result. These data indicated that lncRNA-ROR aggravated H/R-induced cell injury by decreasing cell viability and increasing apoptosis.

### lncRNA-ROR mediated myocardial H/R by regulating p38/MAPK pathway

As shown in Figure 4A and B, phosphorylation of ERK and p38 were significantly up-regulated after treatment of H/R in both H9c2 cells and HCM. Overexpression of lncRNA-ROR further increased H/R-induced activation of phosphorylation of ERK and p38. However, inhibition of lncRNA-ROR abolished the activated effect on H9c2 cells and HCM. These data indicated that lncRNA-ROR might regulate cell growth and induce apoptosis via activation of p38/MAPK signal pathway. The results showed that overexpression of lncRNA-ROR synergistically facilitated H/R-induced the activation of p38-MAPK pathway.

**Figure 4.** lncRNA-ROR mediated myocardial hypoxia/reoxygenation (H/R) by regulating the p38/MAPK pathway. H9c2 cells and human cardiomyocytes (HCM) were transfected with lncRNA-ROR overexpression vector (lncRNA-ROR) and inhibition vector (si-lncRNA-ROR). After H/R treatment for 24 h, (*A*) the protein levels of ERK and p38 were examined by western blot and (*B*) the mRNA expressions of ERK and p38 were determined by qRT-PCR. Data are reported as means±SE. *P<0.05, **P<0.01 (ANOVA).

### Inhibitor of p38/MAPK (SB203580) alleviated lncRNA-ROR-induced cell injury

To further explore the effect of p38/MAPK on cardiomyocytes injury, SB203580 (10 μM) was used to inhibit p38/MAPK expression. The results showed that SB203580 increased lncRNA-ROR-induced cell viability at 24, 48, and 72 h after treatment of H/R in H9c2 cells and HCM (Figure 5A). However, addition of SB203580 significantly decreased cell apoptosis and the cell rate in normoxia, H/R, H/R+lncRNA-ROR, and H/R+lncRNA-ROR+SB203580 were 17.9% (P<0.01), 22.5% (P<0.05), 27.6, and 23.1% (P<0.01) in H9c2 cells, and 4.48% (P<0.001), 13.2% (P<0.01), 17.8, and 14.9% (P<0.01) in HCM (Figure 5B).

**Figure 5.** Inhibitor of p8/MAPK (SB203580) alleviated lncRNA-ROR-induced cell injury. H9c2 cells and human cardiomyocytes (HCM) were transfected with lncRNA-ROR overexpression vector (lncRNA-ROR) and inhibition of p8/MAPK (SB203580, 10 μM). After hypoxia/reoxygenation (H/R) treatment for 24 h, (*A*) cell viability, (*B*) apoptosis, and (*C*) and (*D*) apoptosis-related factors Bax, Bcl-2, cytochrome C, Smac/Diablo, cleaved-caspase-3, and cleaved-caspase-9 were measured by MTT, flow cytometry, qRT-PCR, and western blot, respectively. GAPDH served as the internal control. Data are reported as means±SE. *P<0.05, **P<0.01, ***P<0.001 (ANOVA).

Similarly, SB203580 rescued apoptosis-related factors expressions. As shown in Figure 5C and D, SB203580 down-regulated Bax, cytochrome C, Smac/Diablo, cleaved-caspase-3 and cleaved-caspase-9 expressions, but up-regulated Bcl-2 expression in H9c2 cells and HCM (P<0.05). These data indicated that SB203580 could rescue lncRNA-ROR-induced cell viability and apoptosis in H9c2 cells and HCM.

### lncRNA-ROR promoted ROS production in H9c2 cells

A recent study demonstrated that p38 and ERK were activated by oxidative stress. Therefore, we examined the levels of intracellular ROS production in H9c2 cells. As shown in Figure 6A, H/R treatment significantly enhanced the level of ROS formation, and the effect was further promoted by overexpression of lncRNA-ROR (P<0.05 or P<0.01). However, suppression of lncRNA-ROR reversed the result (P<0.01). To further explore the source of ROS, MitoSOX Red was used to measure mitochondria ROS production. In Figure 6B, the ROS in mitochondria was significantly increased in H/R treatment condition (P<0.05). Overexpression of lncRNA-ROR further promoted mitochondria ROS production (P<0.05). However, the promoting effect were declined by lncRNA-ROR suppression (P<0.05). These results were similar with intracellular ROS production.

**Figure 6.** lncRNA-ROR promoted reactive oxygen species (ROS) production in H9c2 cells. H9c2 cells were transfected with lncRNA-ROR overexpression vector (lncRNA-ROR) and inhibition vector (si-lncRNA-ROR). After hypoxia/reoxygenation (H/R) treatment for 24 h, (*A*) intracellular ROS production was analyzed by H2DCF-DA in H9c2 cells; (*B*) mitochondria ROS production was detected by MitoSOX Red assay; (*C*) the activity of NADPH oxidase was measured by chemiluminescence assay; (*D*) the protein level of NOX2 was examined by western blot. Data are reported as means±SE. *P<0.05, **P<0.01 (ANOVA).

NADPH oxidase plays a crucial role in ROS production, and NOX2 was an important member of the NADPH oxidase family. Therefore, NADPH oxidase activity and NOX2 protein level were examined in H9c2 cells. As revealed in Figure 6C, lncRNA-ROR overexpression enhanced H/R-induced NADPH oxidase activity (P<0.05). In contrast, lncRNA-ROR suppression decreased NADPH oxidase activity (P<0.05). Western blot results displayed that the protein level of NOX2 was increased by H/R treatment, and further enhanced by lncRNA-ROR overexpression. However, lncRNA-ROR suppression reduced NOX2 protein level (Figure 6D). These data revealed that lncRNA-ROR could promote ROS formation in H9c2 cells.

## Discussion

According to World Health Organization estimates, coronary heart disease is the leading cause of death and about 17.5 million people died from cardiovascular disease in 2012 (18). The effects of coronary heart disease are usually caused by the detrimental effects of acute myocardial I/R. The process of myocardial I/R can induce its cell damage and death (19). Since the underlying mechanism of the myocardial I/R injury is unclear, cardiovascular disease remains a leading cause of hospitalization and death globally (20). Therefore, in the present study, we explored the functional role of lncRNA-ROR in myocardial I/R injury. Our results showed that high expression of lncRNA-ROR was observed in I/R patients and in H/R treatment of H9c2 cells and HCM. Moreover, lncRNA-ROR overexpression further increased LDH, MDA, SOD, and GSH-PX releases in H/R treatment H9c2 cells and HCM. The findings suggest that lncRNA-ROR may aggravate H/R-induced myocardial damage.

Recent studies have suggested the critical role of lncRNAs in the regulation of gene expression, which are shown to play an important role in the pathogenesis of cardiovascular diseases (21,22). In another study, it was shown that lncRNA had a protective function for heart from pathological hypertrophy by interfering with the binding of a chromatin remodeling factor Brg1 to chromatinized DNA targets (23). There are several indications that lncRNAs may function as pro-apoptotic or anti-apoptotic regulators (24). Apoptosis plays a crucial role in myocardial I/R (25). In ischemically damaged tissues, activation of pro-death Bcl-2 proteins such as Bax, Bak, Bid, Puma, and BNIP3 and their upregulation, translocation, and integration into mitochondria have been reported (26 [Bibr B27]–28). However, many of these proteins are redox sensitive, which is supported by the fact that ischemia alone is not sufficient for Bcl-2 protein activation and that reperfusion is required (29,30). Both pro- and anti-apoptotic Bcl-2 proteins regulate Ca^2+^ homeostasis, which influences I/R injury (31). Our results were in line with these findings, which showed that due to overexpression of lncRNA-ROR the level of expression of Bcl-2 was decreased, which in turn led to a higher apoptosis rate. Furthermore, overexpression of lncRNA-ROR further increased the level of expression of Bax proteins. These findings indicated that lncRNA-ROR increased cardiomyocyte apoptosis.

To further illustrate the underlying molecular mechanism for apoptosis, which is mediated by lncRNA-ROR, MAPKs such as p38 and ERK were measured. Several studies have indicated that activation of p38 occurs during I/R (32,33), whereas inhibition of p38 has shown reduction in I/R-induced cell death (34,35). We observed that lncRNA-ROR mediated myocardial H/R by regulating the p38/MAPK pathway. This was further proved by the impact of addition of p38 inhibitor (SB203580) to the H9c2 cells. It was observed that SB203580 could rescue lncRNA-ROR-induced cell viability, expression of Bax and Bcl-2, and reduce apoptotic cells rate. These findings are similar to the results obtained in other conditions such as renal I/R injury cells (34), brain cells (35), and chronic myelogenous leukemia K562 cells (36).

Recent studies have demonstrated that ROS is closely related to diverse signal pathways including p38/MAPK (37). Moreover, the production of ROS has been proven to be involved in regulation of myocardial I/R injury (38). In a recent study, Kim et al. (39) demonstrated that PICOT alleviated myocardial I/R injury via decreasing intracellular levels of ROS. Furthermore, mitochondrial and NADPH oxidase are important sources of ROS, and the NADPH oxidase family member of NOX2 exerted an important role in ROS production (40). Based on these studies, we further explored the effect of lncRNA-ROR on ROS formation in myocardial I/R injury. We found that lncRNA-ROR overexpression significantly increased the production of intracellular ROS and mitochondrial ROS. Moreover, the NADPH oxidase activity and NOX2 protein level were also promoted by lncRNA-ROR overexpression in H9c2 cells. These data indicated that lncRNA-ROR-promoted myocardial I/R injury might be associated with the induction of ROS generation. Further studies still need to clarify the hypothesis.

In conclusion, we have shown that lncRNA-ROR plays a crucial role in myocardial I/R injury by regulation of the p38/MAPK signal pathway. Our results suggested that lncRNA-ROR might be an important therapeutic target for myocardial I/R injury and this finding may help in the development of a new strategy for the treatment of myocardial I/R injury.
